# The Relationship between Meniere's Disease and Acute Low-Tone Sensorineural Hearing Loss

**DOI:** 10.1155/2022/4217131

**Published:** 2022-07-07

**Authors:** Yuemei Li, Zhe Lv, Haixia Han, Xiaofang Jia, Lijiao Guo

**Affiliations:** ^1^Department of Vertigo Specialty, The Fourth Central Hospital of Baoding City, Baoding, China; ^2^Department of Otolaryngology, The Second Hospital of Hebei Medical University, Shijiazhuang, China

## Abstract

**Objective:**

To analyse the vestibular function characteristics of patients with Meniere's disease and acute hypophonic sensorineural hearing loss in order to find more reliable and objective ancillary tests that will reduce misdiagnosis and missed diagnoses.

**Methods:**

From January 2021 to December 2021, 60 healthy adults who underwent physical examination in our hospital were included in the control group, 60 patients with Meniere's disease were included in Study Group A, and 60 patients with acute low-tone sensorineural hearing loss were recruited in Study Group B. All participants underwent the caloric test (CT), video-head impulse test (vHIT), headshaking test (HST), and vestibular-evoked myogenic potential (VEMP) testing, which includes ocular vestibular-evoked myogenic potential (oVEMP) and cervical vestibular-evoked myogenic potential (cVEMP).

**Results:**

Statistical analyses of unilateral weakness and directional preponderance (DP) in the two groups of patients found no significant differences between the two groups (*P* > 0.05). There was no statistically significant difference in the abnormal rate of vHIT and HST results between the two study groups (*P* > 0.05). There was no significant difference in the wave latencies, interwave intervals, and amplitudes of cVEMP and oVEMP, among the three groups (*P* > 0.05).

**Conclusion:**

This study found that factors affecting CT, vHIT, HST, and VEMP results included age, head posture and position during testing, stimulus type, manipulation method, and control of muscle tone, and also those that are related to the testing instrument, statistical software, and manipulation procedures, resulting in different excitation rates and testing parameters. The small sample size prevented a comprehensive assessment of the differences in vestibular function between patients with Meniere's disease and acute hypotonic sensorineural hearing loss, and a larger sample size will be investigated in the future to provide useful insight into the diagnosis, treatment and differentiation of Meniere's disease, and acute hypotonic sensorineural hearing loss.

## 1. Introduction

Meniere's disease, also known as idiopathic endolymphatic hydrops, is a disease of the inner ear characterised by idiopathic membranous vagal hydrops involving the auditory and vestibular end organs, with the main clinical manifestations being recurrent episodes of vertigo, undulating hearing loss, tinnitus, and ear swelling [1, 2]. With the accelerated pace of life in modern society, increased work pressure, and deterioration of the living environment, Meniere's disease shows a trend of gradual aggravation [3]. In recent years, there has also been an increasing trend in the incidence of acute low-pitched sensorineural hearing loss of unknown aetiology, with the possible pathogenesis being an accumulation of lymphatic fluid in the cochlea [4]. Its clinical features differ from those of idiopathic sudden sensorineural hearing loss and Meniere's disease. The disease frequently recurs and rarely progresses to Meniere's disease [5]. Currently, the clinical diagnosis of both disorders is made primarily by the patient's clinical symptoms and audiological examination. However, due to the subjective nature of the diagnosis and the similarity in clinical presentation and audiometric findings between early Meniere's disease and acute hypophonic sensorineural hearing loss, the rate of misdiagnosis and missed diagnosis is high. Therefore, exploring more reliable and objective ancillary tests to diagnose and differentiate between these two disorders has become an urgent need for clinical diagnosis [6]. Vestibular function tests are qualitative or quantitative assessments of the physiological function of the vestibular system through specific spontaneous or evoked tests, aiming to clarify the laterality and location of lesions and to understand the degree of impairment of vestibular nervous system function, which are essential for the clinical diagnosis and treatment of vertigo and balance disorders.

The caloric test (CT), the headshaking test (HST) [7], and the video-head impulse test (vHIT) refer to low-frequency (≤0.03 Hz), medium-frequency (1–2 Hz), and high-frequency (2–5 Hz) testing of the vestibular semicircular canal, respectively. The vestibular myogenic evoked potential is what is used to evaluate the function of the utricle and saccule. It is a vestibularly evoked myogenic potential recorded on the surface of muscles such as the sternocleidomastoid and ophthalmic muscles in the presence of strong short acoustic stimulation. Of the vestibular-evoked myogenic potentials (VEMP), the ocular vestibular-evoked myogenic potential (oVEMP) reflects the function of the superior vestibular nerve and the utricle, while the cervical vestibular-evoked myogenic potential (cVEMP) reflects the function of the inferior vestibular nerve and the saccule. In recent years, the presence of vestibular damage in patients with Meniere's disease and acute low-frequency deafness with similar frequency characteristics of cochlear damage has captured great academic attention. Nevertheless, there are few studies on the comprehensive and objective vestibular multiband loss characteristics of Meniere's disease and acute low-tone sensorineural hearing loss. Accordingly, this study analyses the frequency characteristics and sensitivity of the caloric test, HST, vHIT, and VEMP in identifying vestibular function impairment in patients with Meniere's disease and acute low-tone sensorineural hearing loss, to investigate the diagnosis and differentiation of the two diseases and provide more comprehensive data for improving the relevance of vestibular function measurements and the study of its pathological mechanisms.

## 2. Participant and Methods

### 2.1. Participants

From January 2021 to December 2021, 60 healthy adults who underwent physical examination in our hospital were included in the control group, 60 patients with Meniere's disease were included in Study Group A, and 60 patients with acute low-tone sensorineural hearing loss were recruited in Study Group B. All participants in the experimental group had unilateral ear onset. The study was approved by the ethics committee of the Fourth Central Hospital of Baoding City, No. 273791–14, and all participants provided written informed consent.

#### 2.1.1. Inclusion Criteria

Control group: the participants had no previous history of deafness, ear disease, and vertigo with the examination results of normal otoscopy, pure tone audiometry, and acoustic impedance.

Study Group A: ① Patients with episodes greater than 20 minutes/time, at least 2 episodes, frequently accompanied by autonomic dysfunction, balance disorders, but no impairment of consciousness; ② with fluctuating hearing loss, mostly low-frequency hearing loss in the early stage, with hearing loss aggravating as the disease progressed; with at least 1 pure tone audiometry result of sensorineural hearing loss and the potential occurrence of auditory resonance; ③ with tinnitus and a feeling of fullness in the ear; and ④ with vertigo induced by other diseases, such as benign paroxysmal positional vertigo, sudden deafness, and the inadequate blood supply to the vertebrobasilar artery and intracranial occupying lesions.

Study Ggroup B: ① With the acute onset of sensorineural hearing loss (onset to clinic visit within 14 days); ② with mean PTT threshold at low frequencies (125, 250, 500 Hz)≥30 dBHL and mean PTT threshold at high frequencies (2.4.8 kHz)≤20 dBHL; ③ without vertigo and balance disorders, fluctuating hearing changes, spontaneous nystagmus, and history of vertigo attacks; ④ with normal auditory brainstem response (ABR) results; ⑤ without recurrent attacks of symptoms in the recent past; and ⑥ with undefined aetiology by clinical and imaging examinations.

### 2.2. Vestibular Function Testing

#### 2.2.1. Caloric Test

The test apparatus is the Denmark International Hearing EyeSeeCam vestibular function tester, and before the test, the subjects were given precautions of the test for better patient cooperation. The external auditory canal and tympanic membrane were routinely examined to remove cerumen before the examination to exclude otitis media and tympanic membrane perforation. The patient is placed in a supine position, wearing a nystagmus observation eye patch, and hot and cold air (24°C and 50°C, respectively) is instilled into both ears at 8 mL in 1 minute, with the nozzle as close to the tympanic membrane as possible to achieve maximum stimulation. The next instillation was performed only after the patient's nystagmus stopped, and the vertigo sensation disappeared. The examination was suspended if the patient showed signs of vomiting, and the next perfusion stimulation was performed after the patient recovered. The nystagmus viewer recorded and analysed postperfusion nystagmus, and a value of greater than 20% of the hemiplegia (CP) on one side was considered abnormal.

#### 2.2.2. vHIT

The test apparatus is the Denmark International Hearing EyeSeeCam vHIT, and before the test, the subjects were given precautions of the test for better patient cooperation. With the patient in a sitting position and wearing the test eye patch, the examiner stood behind the patient and held the subject's head with both hands, and turned the head within a small range in the corresponding plane to test the corresponding semicircular canal: the horizontal semicircular canal was tested by turning the head from side to side; the right posterior and left anterior semicircular canal function was tested by turning the head right 30–45° in the sagittal plane; the left posterior and right anterior semicircular canal function was tested by turning the head left 30–45° in the sagittal plane. Each plane was tested 15–20 times, and the computer automatically calculated the average value of gain and the presence of sweeping waves (including hidden sweeping waves and dominant sweeping waves). The gain of the horizontal semicircular canal of less than 0.8, the gain of the upper/posterior semicircular canal of less than 0.7, and more than half of the head impulse tests with invisible or dominant sweeping waves were considered abnormal.

#### 2.2.3. HST

With the patient in a seated position at a 30° forward tilt with a video eye patch, the patient kept the eyes open and turned the 30 times with an amplitude of 20° to 30° on the vertical axis of the head. Before the start of HST, the spontaneous nystagmus was recorded for 30 s in the fixation and non-fixation states, and after the cessation of headshaking, the headshaking nystagmus (HSN) was recorded for at least 30 s. The presence of at least five consecutive nystagmuses with nystagmus intensity greater than 2°/s after headshaking was considered positive for HST.

#### 2.2.4. VEMP

The instrumentation is based on the German Keypoint 9033A07 EMG/evoked potentials instrument.

Ocular vestibular-evoked myogenic potential (oVEMP) : The subject is placed in a supine position, the local skin (where the electrodes are placed) is cleaned, the recording electrode is located approximately 1 cm below the midpoint of the inferior orbital rim, the reference electrode is located 1.5–2.0 cm below it, and the ground electrode is located between the eyebrows with an interpolar resistance of less than 5 kΩ. The subject's eyes are gazed upwards at approximately 30° directly above the midline during the test. The waveform of the oVEMP is recorded at the inferior orbital rim of the contralateral eye as a signal in response to this ear stimulus. A stimulus of 100 dBnHL was used to evoke a normal waveform, and the stimulus intensity was gradually decreased in 5-dBnHL intervals until the minimum stimulus intensity at which a response occurred was recorded, which was considered to be the air-conduction oVEMP threshold. A good repetition of the typical waveform complex at the time of recording the threshold was considered a marker of waveform emergence, and the disappearance of the test repetition after 3 stimulations at a specific intensity was considered a marker of response disappearance.

Cervical vestibular-evoked myogenic potential (cVEMP): The subject is placed in a supine position, the skin is cleaned before placement of the electrodes, the recording electrodes are located in the middle of the sternocleidomastoid muscle on both sides, the reference electrodes are placed symmetrically on the surface of the sternocleidomastoid joints on both sides, the ground electrode is located between the eyebrows, and the interpolar resistance is less than 5 kΩ. During the test, the subject's head is slightly raised to maintain tension in the sternocleidomastoid muscle and the head is always in the midline of the body. The cVEMP waveform was recorded on the surface of the ipsilateral sternocleidomastoid muscle as a signal of the response of that ear to the stimulus. Thresholds were defined in the same way as the oVEMP thresholds were determined above.

The oVEMP/cVEMP waveforms were recorded at 100, 95, 90, 85, 80, and 75 dB of nHL acoustic stimulation, and the nI latency, pI latency, nI-pI interwave period, and amplitude were measured. oVEMP latency is the duration (ms) between the start of the test and the nI and pI wave apexes, and interwave period is the duration (ms) between the nI and pI wave apexes. The amplitude is the vertical distance between the nI and pI wave vertices (*μ*V). cVEMP latency is the duration between the test onset and the pI and nI wave vertices (ms), the interwave period is the duration between the pI and nI wave vertices (ms), and the amplitude is the vertical distance between the pI and nI wave vertices (*μ*V). AR values are calculated (using the nI latency as an example). ARr = (right ear nI − left ear nI)/(right ear nI + left ear nI) × 100%. The AR value varies from 0 to 1. The closer to 0, the better the interaural symmetry, and the closer to 1, the worse the interaural symmetry.

### 2.3. Statistical Analysis

SPSS 26.0 software was used for data analysis. The abnormality rates of the calorie test, HST, vHIT, and VEMP test were analysed for each group of participants, and these rates were compared by ANOVA or Kruskal–Wallis statistical assessment. Differences were considered statistically significant at *P* < 0.05.

## 3. Results

### 3.1. Baseline Data

Baseline data for the control group (27 males, 33 females, aged 28–58 years, mean age [40.17 ± 3.39] years) and Study Group A (29 males, 31 females, aged 30–59 years, mean age [41.08 ± 3.84] years, 36 cases of left ear onset and 24 cases of right ear onset) and Study Group B (30 males, 30 females, aged 29–60 years, mean age [41.77 ± 4.13] years, 40 cases in the left ear and 20 cases in the right ear) were not statistically significant (*P* > 0.05).(*P* > 0.05).

### 3.2. Caloric Test

From the CT findings, the number of patients with unilateral weakness in Study Group A was 42 (70.00%) and DP was 37 (61.67%); the number of patients with unilateral weakness in Study Group B was 40 (66.67%) and DP was 35 (8.33%). Statistical analyses of unilateral weakness and DP in the two groups of patients by Fisher's exact test found no significant differences between the two groups (*P* > 0.05) (Table 1).

### 3.3. vHIT and HST

The number of people with vHIT was 17 (28.33%), and the number of people with HST was 0 (0.00%) in Experimental Group A. The number of people with vHIT was 13 (21.67%), and the number of people with HST was 3 (5.00%) in Experimental Group A. There was no statistically significant difference in the abnormal rate of vHIT and HST results between the two study groups (*P* > 0.05) (Table 2).

### 3.4. VEMP

There was no significant difference in the wave latencies, interwave intervals, and amplitudes of cVEMP and oVEMP, among the three groups (*P* > 0.05) (Tables 3 and 4).

## 4. Discussion

Meniere's disease is a common otogenic vertigo disorder with the main clinical manifestations being recurrent episodes of vertigo, fluctuating hearing loss, tinnitus, and a feeling of fullness in the ear. It may affect between 10 and 157 people per 100,000 and is more common in women than in men (a ratio of approximately 1.3 : 1), with a high prevalence between the ages of 40 and 60 years and a prevalence of approximately 3% in children [8, 9]. The main recognised pathogenetic mechanisms include mechanical obstruction of the endolymphatic vessels and impaired endolymphatic absorption, the immune response theory, and the inner ear ischaemia theory. Acute hypotonic sensorineural hearing loss is a syndrome with a distinctive clinical and auditory presentation, with ear congestion as the main symptom [10, 11], an elusive cause, and the development of Meniere's disease if not treated promptly. It was suggested [12] that the disease is related to endolymphatic hydrops, and patients with acute low-tone sensorineural hearing loss are often associated with vestibular impairment regardless of the presence of vertigo. At present, the diagnosis of the two diseases mainly relies on the typical clinical manifestations and audiological test results. However, the same pathogenesis and similar hearing test results complicate the differentiation between them. It has been shown that the otolithic functional examinations are different between the two diseases, but other vestibular function tests have been rarely studied in their differentiation. The organ responsible for vestibular function, called the vestibular apparatus, is located in the inner ear and consists of three semicircular canals (the external, superior, and posterior semicircular canals), the utricle, and the saccule. Each of the utricle and saccule contains an otolithic apparatus. These are the vestibular end receptors, and there is a lack of convenient and practical monitoring techniques that can measure all vestibular endings receptors.

The heat test is a hydrodynamic response in which cold or hot water or air is instilled into the external auditory canal and the temperature of the water or air is conducted through the tympanic membrane to the inner ear, causing thermal expansion and contraction of the endolymph [13]. It can detect bilateral horizontal semicircular canals separately to identify the side of the lesion, but it only examines the function of the ultra-low-frequency region (≤0.03 Hz) of the horizontal semicircular canals [14]. The HST can detect the mid-frequency region (1–2 Hz) of the semicircular canals by observing the direction of nystagmus after shaking the head [15], which is highly sensitive and easily accepted by patients. It has been shown that the combined application of low-frequency calorimetry and mid-frequency headshaking nystagmus can be complementary in the testing of horizontal semicircular canal function. vHIT uses high-frequency and natural passive head-turning stimuli to objectively record head and eye movements (3 pairs of semicircular canal VOR gain values and corresponding 3 gain asymmetry values) and to test 6 semicircular canal high-frequency dynamic functions (2–5 Hz) and horizontal semicircular tube function and the vertical semicircular tube function. The vHIT has been shown to improve the detection rate in patients with peripheral vertigo and is useful for the identification of peripheral vertigo [16, 17]. Vestibular-evoked myogenic potential (VEMP) testing [18] is a noninvasive and simple technique for detecting otolithic vestibular function by evoked potentials generated after the stimulation of the otolithic apparatus by bone-conducted vibration or air-conducted sound. Acoustic stimulation-evoked cervical muscle evoked myogenic potentials (cVEMP) have been used as an objective clinical test for the saccule-subventricular nerve afferent pathway, and the ocular vestibular-evoked myogenic potential (oVEMP) can reflect the function of the superior vestibular nerve and the utricle. It has been suggested [19] that the combination of vestibular tests of oVEMP and cVEMP shows great potential for the examination of the vestibular otolithic conduction pathway, providing new approaches to diagnosing vestibular disorders and exploring the status of the otolithic apparatus. Due to the frequency limitations of all current vestibular assessment techniques, it is essential to combine multifrequency detection techniques to assess vestibular function with more reliable results [20].

The diagnosis of Meniere's disease in Chinese medicine emphasises vertigo in the ear, either due to the weakness of the internal organs, loss of nourishment in the inner ear, or overflow of phlegm and water-dampness in the inner ear [21]. The actual symptoms are paroxysmal vertigo and tinnitus, repeated rotation of vision, head swelling and pain, or faintness and heaviness, irritability, distension in the chest, nausea and vomiting, lack of desire to eat and drink, red tongue, thick and greasy tongue coating or puffy yellow, and a strong or slippery pulse [22]. The deficiency symptoms are occasional dizziness and dizziness, easily recurring or aggravated by exertion, palpitations with little sleep, often with tinnitus, and a pale tongue with a thin pulse as the main evidence [23]. Acupuncture, cupping, massage and tui-na can be used to relieve Meniere's disease, with some effect, but it is slow compared to Western medicine. In the case of acute bass sensorineural hearing loss, TCM considers qi stagnation and blood stasis to be the most important cause in the development of the disease [24]. Many practitioners believe that blood stasis in the ears will eventually occur and that the various forms of violent deafness can often be intermingled with or transformed into blood stasis in the ears, which has been documented as the pathological basis of acute bass sensorineural hearing loss and is central to the development of acute bass sensorineural hearing loss and is always present throughout the process [25]. The use of TCM for the treatment of ALHL can combine various therapeutic methods and complement each other to regulate the functions of the internal organs and promote the body's self-healing, which can not only improve the patient's hearing, but also significantly improve the accompanying symptoms, reduce the patient's distress, and improve the patient's quality of life [26]. Therefore, Chinese medicine can be used to diagnose and treat the two diseases in combination with Western medicine.

This study found that different testing instruments, statistical software, and operating procedures resulted in different excitation rates and testing parameters. From the CT results, the number of patients with unilateral weakness in Study Group A was and the number of patients with DP was more than that in Study Group B. And after the statistical analysis of unilateral weakness and DP in both groups, no statistically significant difference was found between the two groups (*P* > 0.05). The number of vHIT was greater in group A than in group B, but the number of the HST was less than that in group B. However, there was no statistically significant difference in the rate of abnormal vHIT and HST results between the two study groups (*P* > 0.05). The differences in wave latency, interwave interval, and amplitude of cVEMP and oVEMP between the three groups were not statistically significant (*P* > 0.05). In addition, factors influencing the results of CT, vHIT, HST, and VEMP may include age, head posture and position at the time of testing, type of stimulation, method of manipulation, and control of muscle tone.

The small sample size prevented a comprehensive assessment of the differences in vestibular function between patients with Meniere's disease and acute hypotonic sensorineural hearing loss, and a larger sample size will be investigated in the future to provide useful insight into the diagnosis, treatment, and differentiation of Meniere's disease and acute hypotonic sensorineural hearing loss.

## Figures and Tables

**Table 1:** Comparison of caloric test results [n(%)].

Comparison	n	Unilateral weakness	DP
Study Group A	60	42 (70.00)	37 (61.67)
Study Group B	60	40 (66.67)	35 (58.33)
Control group	60	0 (0.00)	4 (6.00%)

The number of patients with unilateral weakness in Study Group A was 42 (70.00%), and the number of DP was 37 (61.67%); the number of patients with unilateral weakness in study B was 40 (66.67%), and the number of DP was 35 (8.33%).

**Table 2:** Comparison of vHIT and HST results [n(%)].

Groups	n	vHIT	HST
Study Group A	60	17 (28.33)	0 (0.00)
Study Group B	60	13 (21.67)	3 (5.00)
Control group	60	0 (0.00%)	0 (0.00)

In Experimental Group A, the number of vHIT was 17 (28.33%), and the number of HST was 0 (0.00%); in Experimental Group A, the number of vHIT was 13 (21.67%), and the number of HST was 3 (5.00%).

**Table 3:** Comparison of cVEMP waveform parameters.

Groups	n	Elicitation rate [n(%)]	PI latency (ms, ±*s*)	NI latency (ms, ±*s*)	Interwave interval (ms, ±*s*)	Amplitude (*μ*V, ±*s*)	AR (%)
Control group	60	60 (100.00)	16.34 ± 1.27	27.33 ± 1.24	11.21 ± 1.31	360.91 ± 24.37	13.37 ± 2.18
Study Group A	60	44 (73.33)^*∗*^^#^	16.91 ± 1.32	26.91 ± 1.35	10.58 ± 1.18	359.48 ± 31.49	26.61 ± 3.72^*∗*^^#^
Study Group B	60	57(95.00)^*∗*^	16.28 ± 1.18	27.18 ± 1.52	11.24 ± 1.40	361.17 ± 25.87	15.88 ± 2.54

*Note.* ^*∗*^ indicates *P* < 0.05 in comparison with the control group; ^#^indicates *P* < 0.05 in comparison with study Group B.

**Table 4:** Comparison of oVEMP waveform parameters.

Groups	Elicitation rate [n(%)]	PI latency (ms, ±*s*)	NI latency (ms, ±*s*)	Interwave interval (ms, ±s)	Amplitude (*μ*V, ±s)	AR(%)
Control group	57 (95.00)	17.73 ± 1.09	12.34 ± 0.58	5.11 ± 0.84	3.66 ± 3.37	11.54 ± 1.59
Study Group A	46 (76.67)^*∗*^^#^	17.38 ± 1.07	11.76 ± 0.91	4.97 ± 0.79	3.59 ± 2.86	24.38 ± 2.77^*∗*^^#^
Study Group B	56 (93.33)^*∗*^	17.64 ± 0.99	12.08 ± 0.74	4.93 ± 0.75	3.76 ± 3.04	13.72 ± 2.36

*Note.* ^*∗*^indicates *P* < 0.05 in comparison with the control group; ^#^indicates *P* < 0.05 in comparison with Study Group B.

## Data Availability

All data generated or analysed during this study are included in this published article.
